The article "Detection of Diseases Using Machine Learning Image Recognition Technology in Artificial Intelligence" was retracted in 2023. Reasons: unreliable results or conclusions; concerns about the data; concerns about the peer review; concerns about the citations.

# Detection of Diseases Using Machine Learning Image Recognition Technology in Artificial Intelligence

**DOI:** 10.1155/2022/5658641

**Published:** 2022-04-13

**Authors:** Jian Huang, Jing Li, Zheming Li, Zhu Zhu, Chen Shen, Guoqiang Qi, Gang Yu

**Affiliations:** ^1^Department of Data and Information, The Children's Hospital Zhejiang University School of Medicine, Hangzhou 310052, China; ^2^Sino-Finland Joint AI Laboratory for Child Health of Zhejiang Province, Hangzhou 310052, China; ^3^National Clinical Research Center for Child Health, Hangzhou 310052, China; ^4^Polytechnic Institute, Zhejiang University, Hangzhou 310052, China

## Abstract

With the continuous development and improvement of artificial intelligence technology, machine learning technology has also been extensively developed, which has promoted the development of computer vision, image processing, natural language processing, and other fields. *Purpose*. This article aims to apply the image processing technology based on machine learning in the detection of childhood diseases and propose the application of image processing technology to the detection of childhood diseases. This article introduces machine learning, image recognition technology, and related algorithms in detail and experiments on image recognition technology based on machine learning. The experimental results show that image recognition technology based on machine learning can well identify white blood cells that are difficult to distinguish with the naked eye, with a recognition rate of up to 90%. Applying image recognition technology based on machine learning in disease diagnosis has greatly improved the level of medical diagnosis.

## 1. Introduction

In a society with rapid development of information, computer technology has begun to approach other traditionally achievable fields. Along with this tendency, many high-tech machines have appeared. At the same time, in order to assist doctors in the treatment, various high-tech appliances have appeared in the traditional medical field. Among them, the emergence of intelligent image recognition technology has reduced a large part of the doctor's energy to analyze the smaller diseased cells in the human body. The design and manufacture of disease diagnosis equipment based on machine learning image recognition technology are becoming more modernized, rationalized, and intelligent. In the medical field, machine-learning-based image recognition technology disease diagnosis equipment uses image collection to analyze and diagnose pathology.

Doctors in major hospitals can quickly diagnose some common diseases based on the image recognition data provided by machine learning, reducing the diagnosis time of the disease, and greatly improving the efficiency and accuracy of the doctor's clinical work. At the same time, image recognition technology based on machine learning can improve the efficiency of diagnosis of intractable diseases. Through the analysis of a large amount of image data and pathological analysis of the symptoms of some diseases, this will provide more valuable rescue time for the rescue of patients, and provide strong data support to improve the efficiency of diagnosis. In addition, it can further reduce the burden on medical personnel. Through image recognition technology, it is also possible to find some cell lesions in the human body that are not easily detectable by doctors, which greatly reduces the incidence of some diseases.

With the development of society, there are more and more researches in related fields such as machine learning. An article published by Byrd et al. describes how to combine sampled curvature information for statistical learning in the Newton-CG method and the limited memory quasi-Newton method. The motivation for this work stems from a supervised machine learning application involving a large number of training points [1]. In the application of machine learning methods, Wang et al. proposed a data-driven, physics-based machine learning method for predicting the difference of RANS modeling Reynolds stress. Using modern machine learning techniques based on random forests, the difference function is first trained using benchmark stream data and then used to predict the Reynolds stress difference in the new stream. This method is used to predict the Reynolds stress in the periodic hill flow using two training stream scenarios with increasing difficulty [2]. Voyant et al. stated in the study that for the good operation of the grid or optimal management of the energy flux entering the Solar System, it is necessary to predict the output power of the Solar System. Before predicting the output of a solar system, the forecast must be focused on solar irradiance. The purpose of Voyant C's research is to outline the use of machine learning methods to predict solar radiation-related content [3]. In the related research on image recognition technology, Shadiev et al. designed a vocabulary learning activity and developed a learning system featuring image-to-text recognition technology to support this activity. He tested the effectiveness of the system in promoting vocabulary acquisition, and also explored learners' views on the tool and the feasibility of the vocabulary learning system [4]. In research on disease diagnosis and prevention, Bomb et al. stated that accidental diagnosis of left ventricular systolic dysfunction is common in clinical practice. In the study, he compared the pressure echocardiogram of the test and found its limitations [5]. He conducted certain research on Internet surveillance systems and updated the current state of knowledge of the event-based Internet biological surveillance system by identifying all systems including current functions. It is hoped that this will help decision-makers determine whether to incorporate the new method into the comprehensive monitoring plan [6]. Hassabis et al. investigated the historical interaction between AI and neuroscience in his research on neuroscience and artificial intelligence. And he emphasized the current progress of AI inspired by neural computing research in humans and other animals [7]. In the research of these researchers, most of them have carried out research on the specific application of machine learning and image recognition technology but lack of research on the development process and development direction of machine learning and other technologies. Therefore, this paper provides a detailed introduction to the conceptual development of machine learning and graphics technology.

The innovation of this article lies in the extensive research on machine learning and machine learning-based image recognition techniques. The application of machine-learning-based image recognition technology to the recognition of white blood cells provides a certain basis for the application of machine learning-based image recognition technology to the diagnosis of diseases.

## 2. Image Recognition Technology and Related Methods of Disease Diagnosis

### 2.1. Machine Learning

Machine learning has two forms of learning: supervised learning and unsupervised learning:

1. Supervised learning, that is, providing right and wrong indications during the machine learning process. Usually the data set contains the final result (0, 1). Algorithms allow the machine to reduce errors by itself. This type of learning is mainly applied to classification and prediction. Supervised learning learns a function from a given training data set, and when new data arrive, the result can be predicted based on this function. The training set requirement for supervised learning is to include input and output, which can also be said to be features and targets. Objects in the training set are annotated by humans. Common supervised learning algorithms include regression analysis and statistical classification.
2. Unsupervised learning, also known as inductive learning, uses *K*-means clustering to establish centers and reduces errors through looping and decreasing operations to achieve the purpose of classification.

Machine learning is a technology that combines artificial intelligence and Big Data application technology, and it is also an important field in the rise of high-performance computer systems in the era of Big Data [8]. At present, the theoretical research content of machine learning is very rich, and the development in many fields is getting faster and better, and it has gradually become one of the research hotspots [9]. There are many machine learning applications in daily life, such as Baidu's Baidu intelligent search engine, Huawei's mobile phone language assistant, and Google's Alphago machine intelligence.  Figure 1 shows some specific applications of machine learning in daily life.

The branched convolutional neural network of machine learning can recognize image information. Compared with humans, machine learning has faster data processing speed, the ability to store information, and extract features. Establishing a deep learning model that can handle image recognition and cognitive abilities can effectively improve applications such as massive image classification, image detection and positioning, image-text conversion, and image semantic segmentation, which have far-reaching effects [10].

Artificial intelligence is a branch of computer science that attempts to understand the essence of intelligence and produce a new intelligent machine that can respond in a similar way to human intelligence. Research in this field includes robotics, language recognition, image recognition, natural language processing, expert systems, and so on. Since the birth of artificial intelligence, the theory and technology have become more and more mature, and the application field has also continued to expand. It is conceivable that the technological products brought by artificial intelligence in the future will be the “container” of human intelligence. Artificial intelligence can simulate the information process of human consciousness and thinking. Artificial intelligence is not human intelligence, but it can think like human beings and may surpass human intelligence.

#### 2.1.1. The Framework of Machine Learning

The machine learning algorithm performs a series of preprocessing operations on the initially obtained data and then extracts part of the data from the data generated after the preprocessing program is completed according to the opinions of experts. At the same time, select appropriate data from the data set as the characteristics of the image. After completing a series of operations, the image modeling work is completed by a specific function [11].  Figure 2 shows the framework of machine learning.

#### 2.1.2. Application of Machine Learning in Medicine

1. Disease diagnosis
2. In the field of medical diagnosis and treatment, medical diagnosis is one of the most common medical activities. Medical disease diagnosis also provides a large amount of analytical data for machine learning, which provides conditions for machine learning in the field of medical diagnosis [12]. Machine learning obtains certain data results by sorting out and analyzing a large amount of medical data. Then, a disease diagnosis model is established through machine learning methods, which can provide medical diagnosis assistance to medical diagnosticians [13].  Table 1 shows the application of each model in disease diagnosis.
3. Medical image processing
4. As the work of medical institutions becomes more and more difficult, many diseases cannot be diagnosed by traditional clinical solutions, and can only be judged by CT, RI, and other means, resulting in a large number of medical images [14]. However, under current conditions, a large number of medical workers can only analyze these medical images themselves. As medical staff have too much subjective initiative such as medical quality, knowledge level, and personal ability, it is easy to lead to misunderstanding of medical images, resulting in some wrong diagnosis results [15]. Image processing technology based on machine learning provides a way to effectively avoid the influence of human factors and improve the accuracy of image content interpretation. The application of each model in medical image processing is shown in Table 2.

### 2.2. Image Recognition Technology

Image recognition refers to people's self-judgment and understanding of images. Computer image recognition technology refers to a technology that analyzes and understands image information [16]. Image recognition is a very important step for the computer to process image information. After the image information is correctly identified, the image information can be analyzed and understood [17]. At present, the accuracy rate of machine learning image processing technology exceeds 99%. Although the accuracy rate is very high, it is necessary to go to the hospital for medical treatment when encountering diseases in daily life.

Image recognition techniques may be based on the main features of the image. Each image has its characteristics, such as the letter A has a point, P has a circle, and Y has an acute angle at the center. The research on eye movement in image recognition shows that the line of sight always focuses on the main features of the image, that is, the places where the contour curvature of the image is the largest or the contour direction suddenly changes, and these places have the greatest amount of information. The scanning route of the eye always goes from one feature to another in turn. It can be seen that in the process of image recognition, the perceptual mechanism must exclude the redundant information of the input and extract the key information. At the same time, there must be a mechanism in the brain responsible for integrating information, which can organize the information obtained in stages into a complete perceptual image.

Image recognition means that people's image recognition mainly includes four stages: image information acquisition, image information preprocessing, feature extraction, category, and classification.  Figure 3 shows a flow chart of image information preprocessing.

#### 2.2.1. Digital Image

The objective things in the natural world reflected by the image are a way of expressing objectively reflecting the natural scenery [18]. A digital image can be represented by a matrix F of size *X* ∗ *Y*, where there are *X* pixels in each row and *Y* pixels in each column, so it can be expressed as follows:

(1) $$\begin{array}{c} F\left(a,b\right)=\left[\begin{array}{cccc} F\left(0,0\right) & F\left(0,1\right) & \ldots & F\left(0,Y-1\right)\\ F\left(1,0\right) & F\left(1,0\right) & \ldots & F\left(1,Y-1\right)\\ \ldots & \ldots & \ldots & \ldots \\ F\left(X-1,0\right) & F\left(X-1,1\right) & \ldots & F\left(X-1,Y-1\right) \end{array}\right]. \end{array}$$

In most cases, traditional matrix marks can also be used to represent digital images and pixels.

(2) $$\begin{array}{c} T=\left[\begin{array}{cccc} t_{0,0} & t_{0,1} & \ldots & t_{0,Y-1}\\ t_{1,0} & t_{1,1} & \ldots & t_{1,Y-1}\\ \ldots & \ldots & \ldots & \ldots \\ t_{X-1,0} & t_{X-1,1} & \ldots & t_{X-1,1} \end{array}\right]. \end{array}$$

Among them, *t*_*a*,*b*_=*F*(*a*, *b*).

#### 2.2.2. Image Filtering

Image noise means that various factors in the image hinder the reception of information. In other words, image noise refers to pixels whose gray values differ greatly from the gray values of neighboring pixels, except for boundary lines and details [19].

*(1) Classification of Image Noise*. Based on the relationship between image and signal, image noise is divided into two types: additive noise and multiplicative noise [20]. Additive noise usually means that the relationship between noise and signal is constantly added. Additive noise has nothing to do with useful signals, but it always interferes with useful signals [21]. In general, additive noise obeys Gaussian distribution. In this case, the noisy image g(*a*, *b*) can be expressed as follows:

(3) $$\begin{array}{c} g\left(a,b\right)=p\left(a,b\right)+l\left(a,b\right). \end{array}$$

The noise signal *l*(*a*, *b*) is usually Gaussian noise with an average value of 0. In other words, noise signals are distributed according to the following rules:

(4) $$\begin{array}{c} Z\left[l\left(a,b\right)\right]={\left(2\pi \alpha^{2}\right)}^{-3/2}\exp\left[-\frac{{\left\|l\left(a,b\right)\right\|}_{2}^{2}}{2\alpha^{2}}\right]. \end{array}$$

Additive noise mainly includes channel noise and noise generated by image scanning. Additive noise and signal are independent of each other [22].

The second type is multiplicative noise. Multiplicative noise is caused by random changes in channel characteristics, and mainly appears on the wireless communication transmission channel [23]. This type of noise is related to the signal and only appears when the signal appears on the aforementioned channel and does not interfere with the signal. When the relationship between noise and signal is proportional, the image g(*a*, *b*) with much noise can be expressed as follows:

(5) $$\begin{array}{c} g\left(a,b\right)=p\left(a,b\right)+l\left(a,b\right)*p\left(a,b\right). \end{array}$$

Gaussian noise and solver noise are the two most common types of noise in images [24]:

(1) Gaussian noise: Gaussian noise follows the characteristics of Gaussian distribution, which is characterized by high noise intensity and large density fluctuation range. The image polluted by Gaussian noise not only affects the gray level of each pixel, but also affects the pollution degree of the same gray level [25, 26]. *G* is used to represent the average value, and when *α* is the standard deviation, the probability density function of Gaussian noise is as follows:
  (6) $$\begin{array}{c} M\left(G\right)=\frac{1}{\sqrt{2\pi \alpha }}\exp\left[-\frac{{\left(G-\partial \right)}^{2}}{2\alpha^{2}}\right]. \end{array}$$
(2) Salt and pepper noise: salt and pepper noise is also called impulse noise, and its appearance is random. The gray value of the contaminated pixel is the pixel value near the maximum or minimum value of the image gray value range. The probability density function of salt and pepper noise is as follows:
  (7) $$\begin{array}{c} M\left(G\right)=\left\{\begin{array}{cc} M_{x}, & G=x,\\ M_{y}, & G=y,\\ 0, & \text{other}. \end{array}\right) \end{array}$$
(3) Rayleigh noise: the probability density function of Rayleigh noise is as follows:
  (8) $$\begin{array}{c} M\left(G\right)=\left\{\begin{array}{cc} \frac{2}{y}\left(G-x\right)\exp\left[-\frac{{\left(G-x\right)}^{2}}{y}\right], & G\geq x,\\ 0, & G\leq x. \end{array}\right) \end{array}$$

The mean and variance of the probability density are as follows:

(9) $$\begin{array}{c} \partial =x+\sqrt{\frac{\pi y}{4}},\\ \alpha^{2}=y\frac{\left(4-\pi \right)}{4}. \end{array}$$

*(2) Evaluation Criteria for Filtering Performance*. Generally speaking, there are three considerations for evaluating the effect of a filtered image: the degree of noise attenuation, the degree of edge preservation, and the degree of regional smoothness. In order to evaluate the filtering performance reasonably, people mainly divide the evaluation methods into two types: objective evaluation and subjective evaluation.

Objective evaluation mainly reflects the quality of the filtering performance according to the size of the specific parameters of the filtered image. It mainly includes mean square error (MSE), peak signal-to-noise ratio (PSNR), minimum absolute error (MAE), normalized mean square error (NMSE), and image signal-to-noise ratio improvement factor *R*. The calculation formulas of these evaluation methods are listed below, where *f*(*a*, *b*) represents the gray value of the filtered image, *y*(*a*, *b*) is the gray value of the original image, and the image size is *X* ∗ *Y*:

(i) Mean square error (MSE):
  (10) $$\begin{array}{c} \text{MSE}=\frac{1}{XY}{\sum_{X=0}^{X-1}\sum_{Y=0}^{Y-1}\left[y\left(a,b\right)-f\left(a,b\right)\right]}^{2}. \end{array}$$
(ii) Peak signal-to-noise ratio (PSNR):
  (11) $$\begin{array}{c} \text{PSNR}=10\;\log\frac{255^{2}}{1/XY\sum_{X=0}^{X-1}{\sum_{Y=0}^{Y-1}\left[y\left(a,b\right)-f\left(a,b\right)\right]}^{2}}. \end{array}$$
(iii) Minimum absolute error (MAE):
  (12) $$\begin{array}{c} \text{MAE}=\frac{1/XY\sum_{X=0}^{X-1}\sum_{Y=0}^{Y-1}\left|y\left(a,b\right)-f\left(a,b\right)\right|}{\sum_{X=0}^{X-1}\sum_{Y=0}^{Y-1}\left|y\left(a,b\right)\right|}. \end{array}$$
(iv) Normalized mean square error (NMSE):
  (13) $$\begin{array}{c} \text{NMSE}=\frac{1/XY{\sum_{X=0}^{X-1}\sum_{Y=0}^{Y-1}\left[y\left(a,b\right)-f\left(a,b\right)\right]}^{2}}{\sum_{X=0}^{X-1}\sum_{Y=0}^{Y-1}{\left[y\left(a,b\right)\right]}^{2}}. \end{array}$$
(v) Image signal-to-noise ratio improvement factor *R*:
  (14) $$\begin{array}{c} \text{PSNR}=10\;\log\frac{1/XY{\sum_{X=0}^{X-1}\sum_{Y=0}^{Y-1}\left(f\left(a,b\right)-l\left(a,b\right)\right)}^{2}}{1/XY\sum_{X=0}^{X-1}\sum_{Y=0}^{Y-1}{\left(y\left(a,b\right)-l\left(a,b\right)\right)}^{2}}. \end{array}$$

If the noise is effectively suppressed after filtering, the *R* obtained by the formula is a negative value.

#### 2.2.3. Image Recognition Algorithm

Image recognition belongs to the category of pattern recognition, and its recognition algorithms mainly include template matching, statistical pattern recognition, structural pattern recognition, fuzzy image recognition, and intelligent pattern recognition. The first three algorithms are relatively mature and show good performance in many aspects. They are the basis of image recognition algorithms.

*(1) Statistical Pattern Recognition*. Statistical pattern recognition is the basic process of computer recognition, which is mainly based on mathematical decision theory to establish recognition patterns. This is the method with the smallest classification error. The basic idea is to first discover regularity by performing multiple statistical analyses on the survey object, and then directly or implicitly use various probability density functions and postprobabilities to select and identify the essential characteristics of the images that reflect the classification. This is mainly to use Bayesian rules to solve the problem of optimal classifiers, but the estimation of probability density is a more difficult problem to solve in the implementation process.  Figure 4 shows the implementation process of statistical pattern recognition.

*(2) Structural Pattern Recognition*. Structural pattern recognition is also called grammatical pattern recognition. The basic idea is to use most simple subpatterns to correctly represent complex patterns. It is also possible to split the subpattern into several simple primitive attributes and then convert the complex pattern recognition into a simple primitive identity recognition.  Figure 5 shows the realization process of structural pattern recognition.

#### 2.2.4. Image Feature Analysis Method

Principal component analysis method and linear discriminant analysis method are the most common image feature analysis methods.

*(1) Principal Component Analysis Method*. PCA is a typical feature extraction and data representation technology. The PCA analysis method can effectively extract the most important elements and structures in the data, eliminate useless noise and redundant information, and simplify the original data. Furthermore, the simple meaning behind the cumbersome data is discovered, and it has been widely used in the field of pattern recognition and computer vision. The principle of PCA is as follows:

Assuming that the training sample {*R*1, *R*2,…, *Rn*} is transformed into a one-dimensional vector, there is *R*_*l*_∈*T*^*n*−1^(*l*=1,2,…, *N*), and its vector mean is recorded as $\bar{R}$, let

(15) $$\begin{array}{c} M=\left[r_{1}-\bar{r},r_{2}-\bar{r},\ldots ,r_{n}-\bar{r}\right]\in T^{n*N}. \end{array}$$

Then, the covariance matrix can be expressed as follows:

(16) $$\begin{array}{c} E_{t}=\frac{1}{N}MM^{T}. \end{array}$$

Let the matrix be

(17) $$\begin{array}{c} V_{\text{pca}}=\left[v_{{\text{pca}}_{q}},v_{{\text{pca}}_{2q}},\ldots ,v_{{\text{pca}}_{n}}\right], \end{array}$$

where *v*_pca_*q*__, *v*_pca_2*q*__,…, *v*_pca_*n*__ is the eigenvector of *E*_*t*_.

*(2) Fisher Linear Discriminant Method*. Fisher linear discriminant analysis method is also used to reduce the dimensionality of the data to reduce the complexity of the operation. The basic rule it relies on is that the distribution of samples of different types should be as far as possible, and the distribution of samples of the same type should be as close as possible. Supposing there are *W* images in the training sample set: {*a*_1_, *a*_2_,…, *a*_*n*_}, where *ai* represents a column vector obtained by connecting each column of an image. And divide it into *c* categories, representing *A*_1_, *A*_2_,…, *A*_*c*_, and the dimension of the sample is *d*. The number of samples of class *a*_*i*_ is *W*_*i*_, the sample mean vector of this class *a*_*i*_ and the total mean vector of all samples are

(18) δi=1Wi∑j=iWiaj,aj∈Ai,δ=1Wi∑j=iWiaj.

So the overall dispersion matrix can be calculated as follows:

(19) $$\begin{array}{c} Y_{O}={\sum_{i=1}^{O}\left(a_{i}-\delta \right)\left(a_{i}-\delta \right)}^{O}\\ =\sum_{i=1}^{c}\sum_{a\in A_{i}}\left(a-\delta_{i}+\delta_{i}-\delta \right){\left(a-\delta_{i}+\delta_{i}-\delta \right)}^{O}\\ =\sum_{i=1}^{c}\sum_{a\in A_{i}}\left(a-\delta_{i}\right){\left(a-\delta_{i}\right)}^{O}+\sum_{i=1}^{c}W_{i}\left(\delta -\delta_{I}\right){\left(\delta -\delta_{i}\right)}^{O}\\ =Y_{e}+Y_{u}. \end{array}$$

Suppose the transformation matrix is *K* = [*K*_1_, *K*_2_,…, *K*_*n*_], and the sample {*m*_1_, *m*_2_,…, *m*_*n*_} after the transformation matrix is *H*_1_, *H*_2_,…, *H*_*n*_. Their mean vector and scatter matrix are as follows:

(20) $$\begin{array}{c} {\tilde{\delta }}_{i}=\frac{1}{n_{i}}\sum_{i=1}^{n_{i}}H_{i},\\ \tilde{\delta }=\frac{1}{n_{i}}\sum_{i=1}^{n}H_{i},\\ Y_{e}={\sum_{i=1}^{c}\sum_{H\in H_{i}}\left(H-{\tilde{\delta }}_{i}\right)\left(m-{\tilde{\delta }}_{i}\right)}^{O},\\ Y_{i}=\sum_{i=1}^{c}n_{i}\left(\tilde{\delta }-{\tilde{\delta }}_{i}\right){\left(\tilde{\delta }-{\tilde{\delta }}_{i}\right)}^{O}. \end{array}$$

The dispersion of the sample can be measured by the determinant of the dispersion matrix, and the Rayleigh coefficient can be calculated. By solving the correlation of the Rayleigh coefficients, the solved projection vector and the transformation matrix composed of the projection vector can be obtained.

### 2.3. Childhood Disease Detection

As the age of children continues to grow, the physical and mental health of children is constantly changing. For children, those with insufficient resistance are often susceptible to the interference of some viruses, which can cause some diseases. In the world, children and the elderly are the most vulnerable groups. At present, the diseases that children are most susceptible to can be divided into six categories, as shown in Figure 6.

#### 2.3.1. Common Diseases

1. Respiratory diseases: common respiratory diseases in children mainly include: fever, febrile convulsion, cough, asthma, and so on
2. Intestinal diseases: common intestinal diseases in children include: diarrhea, abdominal pain, and constipation
3. Infectious diseases: the most common infectious diseases in children include: hand, foot, and mouth disease; influenza; measles; and so on. In particular, hand, foot, and mouth disease is the most widely spread of childhood diseases
4. Skin diseases: the most common skin diseases in children include: eczema; hand, foot, and mouth disease; chickenpox; acute rash in children; and so on
5. Oral diseases: the most common oral diseases in children include: bad breath, bottle teeth, thrush, and so on
6. Eye diseases: the most common eye diseases in children include: myopia, strabismus, and allergic conjunctivitis

The most common eye diseases in children include: myopia, strabismus, and allergic conjunctivitis.

#### 2.3.2. Common Disease Diagnosis Methods

1. Acute gastroenteritis: the clinical manifestations are abdominal pain, diarrhea, abdominal distension, middle and upper abdominal tenderness, active bowel sounds, and white blood cells which can be increased by blood analysis.
2. Acute gastritis: it is more common in eating spicy and other irritating food, catching cold, and so on, sudden upper abdominal pain, mainly under the xiphoid process, may be dull pain, colic, distending pain, accompanied by nausea, vomiting, belching, acid reflux, and so on. Gastroscope can find changes such as acute gastric mucosal erosion and redness.
3. Hand, foot, and mouth disease: the clinical manifestations of this disease are complex and diverse. Most patients have mild symptoms, with or without fever, and are mainly characterized by scattered rash or herpes on the feet, mouth, and buttocks; a few patients may have multiple complications; individual critically ill children progress rapidly and may die.

## 3. Application Experiment of Image Recognition Technology Based on Machine Learning in Disease Detection

### 3.1. Cell Recognition Experiment Based on Machine Learning

For high-resolution cell images, white blood cells are segmented based on traditional image recognition algorithms. Then the texture feature, color feature, size and shape and other features are extracted, and then differentiated according to the feature difference of different types of cells. Image preprocessing based on traditional image recognition algorithms is much more complicated. In contrast, image recognition based on convolutional neural networks is not the case. It only needs to include the target map in the training set, and the proportion is relatively large. It has a large tolerance for some background interference, light effects, and so on. Therefore, the use of high-resolution cell images to confirm the reliability and separability of the data set is mainly based on the convolutional neural network algorithm to verify.

First, for high-resolution white blood cell images, a deep network structure is used to learn and train.  Table 3 shows the structure of the convolutional neural recognition network of the color white blood cell map based on the AlexNet network structure.

There is an activation layer behind each convolutional layer, which uses the Relu activation function. After the first two fully connected layers, there is a Dropout layer with a randomness shielding factor of 0.5. This shows that half of the weight parameters of the fully connected layer do not participate in back propagation. As the maximum resolution of the collected white blood cells is 170 × 170 × 3, the input size is 170 × 170 × 3.

After deep network training, learning, and testing, it can be concluded that the data set produced by oneself is separable and the recognition rate is high. However, as the coaxial lensless system collects grayscale images, the color image is converted into a grayscale image, and only the input layer of the network is changed, and the training result of the deep network white blood cell grayscale image can be obtained.

### 3.2. Image Recognition Experiment Based on Machine Learning

Pattern recognition originated in the field of engineering, and machine learning originated in computer science, and the combination of these two different disciplines has brought about the adjustment and development of the field of pattern recognition. Pattern recognition research mainly focuses on two aspects:

1. The study of how objects (including people) perceive objects belongs to the category of cognitive science
2. Under the given task, how to use the computer to realize the theory and method of pattern recognition, these are the strengths of machine learning and one of the contents of machine learning research

Pattern recognition has a wide range of applications, including computer vision, medical image analysis, optical character recognition, natural language processing, speech recognition, handwriting recognition, biometric recognition, document classification, search engines, and so on, and these fields are also machine learning exhibitions skilled arena, so pattern recognition and machine learning are more and more closely related.

In this paper, 100 images related to childhood diseases are selected as the images to be tested, that is, taking 100 children as the research object. Each image is automatically scored using image recognition technology. Finally, the image recognition score is compared with the professional score, and the error of the automatic scoring experiment is statistically analyzed. The experimental results are summarized in Tables 4 and 5.

### 3.3. Recognition Experiment of Low-Resolution Cell Images Based on Machine Learning

Low-resolution cells contain the main features of the cells, and the features of the cells can also be extracted and distinguished through the convolutional neural network under the conditions of sufficient database. Based on the lensless microscopic cell image, the original size of the cell is of low resolution, and it also has diffraction pattern spots, but it is difficult for the human eye to distinguish the diffraction pattern spots.

Low-resolution nondiffraction white blood cell images can be collected by a microscope, which is difficult for the human eye to distinguish. Therefore, the data obtained by down-sampling the labeled high-resolution cell images are used for experiments. First, the data set gradually reduces the resolution image from 170 × 170 high-resolution images, and produces white blood cell data sets with different resolutions. Then choosing the same network and the same training parameters to compare the experimental results.

## 4. Experimental Results of Image Recognition Technology Based on Machine Learning

### 4.1. Experimental Analysis of Cell Recognition Based on Machine Learning

In the cell recognition experiment based on machine learning, experiments were performed on the deep-level network white blood cell color data set and the high-resolution shallow network gray-level white blood cell recognition, respectively.  Figure 7 shows the results of this experiment.

According to Figure 7, it can be concluded that regardless of the white blood cell recognition method, the recognition rate is basically stable above 90%. The recognition rate of deep network on color images is significantly higher than that on gray images. For the phenomenon that the recognition rate of gray images is not high, the main reasons are as follows: First, the network structure is not particularly sensitive to the learning of gray images. Second, the input grayscale image is small, the data dimension is too small, and the features extracted by the deeper network from its learning and training are too detailed, which makes the network's generalization ability weak.

In the experiment of cell recognition based on machine learning, the role of convolutional layer in image recognition in convolutional neural network is also studied.  Figure 8 shows a graph showing the influence of the number of different convolution kernels on the image recognition rate.

It can be concluded from Figure 8 that Alexnet is more sensitive to colors and has poor ability to recognize grayscale images. Lenet5 is more sensitive to grayscale images. For high-resolution grayscale white blood cell images, the network structure should use a shallower network structure. And for the experimental result data set of this experiment, the number of convolutional layers and the number of convolution kernels used should not be too many.

### 4.2. Image Recognition Experiment Based on Machine Learning

In the experiment of image recognition based on machine learning, 100 images related to childhood diseases were tested as images to be tested, and each image was automatically scored using image recognition technology. Finally, the image recognition score was compared with the professional score, and the experimental results were also recorded. According to Tables 4 and 5, the comparison chart of the recognition rate of the two different methods in image recognition in this experiment can be obtained, as shown in Figure 9.

It can be concluded from Figure 9 that the recognition rate of the PCA image recognition method at 0 error is 9% higher than that of the FLD method. However, the recognition error rate of these two methods is much lower than the image recognition error rate of manual recognition.

### 4.3. Recognition Experiment of Low-Resolution Cell Images Based on Machine Learning

According to the data analysis of low-resolution cell image recognition experiments, the recognition success rate of different resolutions in image recognition is obtained.  Figure 10 shows the image recognition rate data graph under different resolutions and different networks.

It can be found from Figure 10 that as the resolution decreases, the recognition rate is slowly decreasing, but it is basically above 90%. But when the resolution is reduced to 15 × 15 size, the recognition rate drops suddenly. At this time, because the cell resolution is too low and too much information is lost, the network cannot identify white blood cells. In the case of low resolution, white blood cells can also learn their characteristics through the neural network and achieve the purpose of classification, but the recognition is only 90%. Moreover, it can be found from Figure 10 that the recognition rate of low-resolution nondiffraction leukocytes can reach 91% with the image recognition technology based on machine learning, and the recognition rate of low-resolution diffracted white blood cell maps can reach about 90%.

## 5. Conclusion

Machine learning is a multifield interdisciplinary subject involving probability theory, statistics, approximation theory, convex analysis, algorithm complexity theory, and other disciplines. It specializes in how computers simulate or realize human learning behaviors to acquire new knowledge or skills, and to reorganize existing knowledge structures to continuously improve their performance. Through the experiments in this article, the following conclusions can be drawn. The image recognition technology based on machine learning analyzes and summarizes the patient's medical record data according to the characteristic value of the disease and supports the classification of various diseases. It can improve the work efficiency of medical staff and at the same time reduce the burden on medical staff. At the same time, image recognition technology based on machine learning can well find hidden diseases that are difficult for doctors to discover during the growth period of children and better protect the growth of children. This technology can help the pharmaceutical industry to improve the quality of medicines, making medicines work faster and have fewer side effects than conventional medicines. The experimental results in this article show that the recognition rate of low-resolution nondiffraction white blood cells has exceeded 90% based on the image recognition technology of machine learning. This is a good way to find out whether there are abnormal white blood cells during the growth of children, which greatly reduces the risk of children suffering from diseases.

## Figures and Tables

**Figure 1:** Application of machine learning in daily life.

**Figure 2:** The framework of machine learning.

**Figure 3:** Image preprocessing flow chart.

**Figure 4:** Flow chart of statistical pattern recognition.

**Figure 5:** Flow chart of structural pattern recognition.

**Figure 6:** Six categories of diseases commonly seen in children.

**Figure 7:** Results of white blood cell recognition rate based on different methods.

**Figure 8:** The influence of the number of different convolution kernels on the image recognition rate: (a) convolution kernel (five) and (b) convolution kernel (six).

**Figure 9:** Comparison of image recognition rates of two different methods.

**Figure 10:** Image recognition rate under different resolutions and different networks.

**Table 1:** Application of each model in disease diagnosis.

Years	Model	Field
2013–2014	SAE, CNN, DBM + SVM	Cancer diagnosis
2014	DBM	Chronic gastritis diagnosis
2014–2015	SAE	AD classification
2015	CNN	Nuclear cataract classification

**Table 2:** Application of each model in medical image processing.

Years	Model	Field
2013	CNN and DBN	Image key point discovery
2013–2014	CNN	Automatic segmentation of medical images
2014	SAE	MRI image reconstruction

**Table 3:** Convolutional neural network structure for high-resolution color white blood cell recognition.

	Input	Conv1	Pool1	Conv2	Pool2	Conv3	Pool3	Fc4	Fc5	Fc6
Fiter size		11 ∗ 11	3 ∗ 3	5 ∗ 5	3 ∗ 3	3 ∗ 3	3 ∗ 3			
Channel	3	96	256	256	256	256	256	4096	4096	3
Strides		3	2	1	2	1	2			
Padding				2		1	1			

**Table 4:** Summary table of PCA method experimental results.

Error distribution value	Quantity	Percentage
0	60	60
−1 to 1	21	21
−2 to 2	9	9
−3 to 3	7	7
−3.5 to 3.5	3	3
Total	100	100

**Table 5:** Summary table of experimental results of the FLD method.

Error distribution value	Quantity	Percentage
0	51	51
−1 to 1	26	26
−2 to 2	10	10
−3 to 3	9	9
−3.5 to 3.5	4	4
Total	100	100

## Data Availability

The data used to support the findings of this study are available from the corresponding author upon request.
